# NEK2 plays an active role in Tumorigenesis and Tumor Microenvironment in Non-Small Cell Lung Cancer

This article has been retracted.

**DOI:** 10.7150/ijbs.59019

**Published:** 2021-05-11

**Authors:** Rui Bai, Cheng Yuan, Wenjie Sun, Jianguo Zhang, Yuan Luo, Yanping Gao, Yangyi Li, Yan Gong, Conghua Xie

**Affiliations:** 1 Department of Radiation and Medical Oncology, Zhongnan Hospital of Wuhan, University, Wuhan, Hubei 430071, China.; 2 Department of Biological Repositories, Zhongnan Hospital of Wuhan, University, Wuhan, Hubei 430071, China.; 3 Tumor Precision Diagnosis and Treatment Technology and Translational Medicine Hubei Engineering Research Center, Zhongnan Hospital of Wuhan University, Wuhan, Hubei 430071, China.; 4 Hubei Key Laboratory of Tumour Biological Behaviors, Zhongnan Hospital of Wuhan University, Wuhan, Hubei 430071, China.; 5 Hubei Cancer Clinical Study Center, Zhongnan Hospital of Wuhan University, Wuhan, Hubei 430071, China.

**Keywords:** NEK2, NSCLC, tumorigenesis, Wnt/β-catenin, tumor microenvironment

## Abstract

Abnormal expression and dysfunction of Never-in-mitosis-A-related kinase 2 (NEK2) result in tumorigenesis. High levels of NEK2 are related to malignant progression, drug resistance, and poor prognosis. However, the relationship between NEK2 levels and the occurrence of non-small cell lung cancer (NSCLC) remains unknown. This study aimed to explore the impacts of NEK2 on the oncogenesis of NSCLC and the tumor microenvironment. Downregulation of NEK2 inhibited A549 and H1299 cell proliferation, migration, and invasion, blocking cell cycle at the G0/G1 phase. Loss of NEK2 inhibited the release of IL-10 from tumor cells, M2-like polarization of macrophages, angiogenesis, and vascular endothelial cell migration. Furthermore, NEK2 deficiency inhibited tumor growth *in vivo*. Taken together, NEK2 knockdown inhibited the occurrence and development of NSCLC, M2 polarization of macrophages, and angiogenesis. The abnormal expression of NEK2 might not only indicate tumor progression and patient prognosis but also serve as a potential molecular therapeutic target with great development prospects.

## Introduction

Lung cancer is a malignant tumor originating from bronchial mucosa epithelium or gland, and it is one of the main causes of cancer-related deaths worldwide. Non-small cell lung cancer (NSCLC) is a common clinical type, accounting for approximately 85% of lung cancer cases 1, 2. Factors including smoking, occupation, environmental exposure, previous chronic lung infections, air pollution, and poverty may be related to a higher prevalence of lung cancer 3, 4. Although research on the characteristics and treatment methods of NSCLC (such as surgery, adjuvant therapy, chemotherapy, radiotherapy, and immunotherapy) has made great progress, the 5-year survival rate in NSCLC patients is still low 5-7.

Never-in-mitosis-A-related kinase 2 (NEK2) is a cell cycle regulatory protein kinase that plays an important role in the mitosis of cells 8. The NEK2 protein has 3 splice isomers with a highly homologous structure 9. The increased expression of NEK2 in malignant tumors was originally discovered in Ewing's tumors 10. Studies have shown that NEK2 is involved in a variety of human cancers, including NSCLC 11, 12, myeloma 13, ovarian cancer 14, breast cancer 15, 16, prostate cancer 17, and colorectal cancer 18. Zhong *et al.* analyzed 270 NSCLC tissues and found that the expression levels of NEK2 were similar to those of 2 known cell proliferation markers, MCM7 and Ki67, which indicates tumor cell proliferation 11. Statistical analysis showed that there was a negative correlation between NEK2 expression levels and the overall survival of patients. Therefore, NEK2 may be an important tumor marker, and its expression levels may predict tumor proliferation and prognosis.

Although immune checkpoint inhibitors such as anti-cytotoxic T lymphocyte-associated protein 4 and anti-programmed cell death protein 1 have shown certain effects in the treatment of lung cancer, only a small number of patients benefit from therapies at the lowest toxic therapeutic dose 19-22. The reason for these results is that lung cancer cells acquire a large number of somatic mutations and various immune evasion mechanisms such as secretion of pro-tumor cytokines, imbalance in antigen expression, and inactivation of T cells 23-26. Current research focuses on the analysis of immune cells in the tumor microenvironment (TME) and their impact on the occurrence of lung cancer.

TME is a unique system composed of malignant tumor cells, tumor-infiltrating immune cells, embryonic cells, glial cells, tumor-associated fibroblasts, cytokines and chemokines secreted by these cells. Various cells in the TME interact and affect each other. Their metabolites are the source of energy supply to each other and mediate the transmission of information between various cells in the TME 27. The interaction between malignant tumor cells and immune cells in TME synergistically promotes tumor development.

Since the role of NEK2 in NSCLC remains unclear, we aimed to evaluate the effect of NEK2 expression on cell proliferation, migration, and invasion. In this study, we demonstrated better prognosis in NSCLC patients with lower NEK2 levels. NEK2 knockdown inhibited NSCLC cell proliferation and epithelial-mesenchymal transition (EMT) via regulating the Wnt/β-catenin signaling pathway. NEK2 deficiency inhibited M2-like macrophages and angiogenesis. These results imply that NEK2 may be a target for lung cancer treatment.

## Materials and methods

### Bioinformatics analysis based on TCGA database

The RNA sequencing datasets of lung cancer and the corresponding clinical information were obtained from The Cancer Genome Atlas (TCGA). After normalization, the differentially expressed genes (DEGs) between lung cancer tissues and normal controls were calculated using the limma package 28 with a cutoff value of |log2FC| > 2 and an adjusted P-value < 0.05. GEPIA (http://gepia.cancer-pku.cn/) was used to analyze differential expression, relationships between NEK2 and clinical stage and survival. The Kyoto Encyclopedia of Genes and Genomes (KEGG) pathway analysis was performed using the cluster Profiler package 29. The cutoff criterion was a P-value < 0.05. Gene Set Enrichment Analysis (GSEA) was downloaded from GSEA HOME and run in a Java environment. Significant gene sets with an FDR < 25% and a nominal P-value < 0.05 were identified.

### Cell culture

We purchased NSCLC cell lines (A549, PC9, H1299, and H1975) from the Type Culture Collection of the Chinese Academy of Sciences (Shanghai, China). We used the RPMI-1640 medium (Hyclone Ltd., USA) supplemented with 10% fetal bovine serum (FBS) (Hyclone Ltd., USA) to culture all cells and maintain the cultured cell lines in a humidified atmosphere containing 5% CO_2_ at 37 °C.

### RNA extraction and qRT-PCR

Total RNA was isolated from cells using TRIzol reagent (Vazyme Ltd., China). We used HiScript® Q RT SuperMix (Vazyme Ltd., China) to transcribe RNA and ChamQTM SYBR® qPCR Master Mix (Vazyme Ltd., China) to perform qRT-PCR. The primer sequences are listed in Table S1.

### siRNA and lentiviral transfection

We transfected NEK2-specific siRNAs or non-specific siRNAs as negative control (NC) synthesized by Shanghai GenePharma Company (Shanghai, China) using the jetPRIME transfection reagent (Polyplus-transfection® SA, France). We used puromycin (Cayman Chemical Ltd., USA) to select stable knockdown cells (successfully transfected with lentiviral-shNEK2) at a concentration of 4 ug/mL for A549 and H1299 cells, respectively. siRNA sequences are listed in Table S2.

### Plasmid vector transfection

Negative control and recombinant plasmid vectors overexpressing NEK2 (GeneCopoeia, USA) were constructed to transfect cells using Lipofectamine 2000 transfection reagent (Invitrogen; Thermo Fisher Scientific, Inc.).

### Cell proliferation assay

Cell Counting Kit-8 (CCK‐8) and colony formation assays were carried out as described previously 30.

### Cell cycle analysis

Cells were treated with the Cell Cycle Staining Kit (MultiSciences Biotech Ltd., China) after washing with cold phosphate-buffered saline. Flow cytometry (Beckman, USA) was used to detect the percentage of cells existing at different cell cycle phases.

### Immunohistochemistry and immunofluorescence

We used antibodies for NEK2, CD163, IL-10, CD31, E-cadherin, Vimentin, and Ki67 (1:100, Proteintech) to incubate specimens at 4 °C overnight, followed by incubation with HRP-labeled secondary antibodies and DAB according to the manufacturer's instructions. Immunofluorescence was performed as previously described 30.

### Transwell assays

A549 or H1299 cells were seeded in the upper chamber of a Transwell plate (Corning Ltd., USA). The lower chamber contained 500 µL of the medium supplemented with 10% FBS. After 48-h incubation, the migrated cells were fixed with formaldehyde and stained with 0.5% crystal violet (Sigma-Aldrich; Merck KGaA).

### Wound healing assays

Transfected cells were seeded in 6-well plates, and later, the cell layer was scratched with a pipette tip. We used the following formula to calculate the migration rate: wound closure (%) = (distance of the initial scratch - distance of the final imaged without cells) / distance of the initial scratch.

### Immunoblotting

We used a 10% SDS-PAGE gel to separate the proteins and transfer them to a PVDF membrane. We used the following antibodies to probe NEK2, p21, p27, CDK2, CDK4, CDK6, cyclinD1, E-cadherin, N-cadherin, Vimentin, MMP9, MMP2, p-GSK3β (Ser9), t-GSK3β, β-catenin, c-Myc, IL-10, and GAPDH at 4 °C for 12 h and incubated with HRP-conjugated secondary antibody for 2 h following detection by chemiluminescence (Bio-Rad Laboratories, Inc., USA). Antibodies used for immunoblotting are listed in Table S3.

### Tube formation assay

Human umbilical vein endothelial cell (HUVECs) (10^4^ cells/well) were seeded in a Matrigel-coated 96-well plate and cultured in a serum-free medium for 6 h. Cells were then cultured with various conditioned media from H1299 and A549 cells for 24 h. Tube length was evaluated from the images using ImageJ software.

### Macrophages generation and differentiation

We treated THP-1 with PMA (Sigma-Aldrich, USA) to generate M0 macrophages. To mimic tumor-associated macrophage (TAM) formation, M0 macrophages were cultured in the conditioned supernatant of lung cancer cells (A549 or H1299) in 6-well plates.

### Xenograft tumor model

All animal experiments were performed according to the guidelines of the Institutional Animal Care and Use Ethical Committee of the Zhongnan Hospital of Wuhan University. The mice purchased from Vital River Laboratory Animal Technology (Beijing, China) were randomly grouped as follows: LV-NC H1299 cells (10^7^), LV-NC H1299 cells (10^7^) and TAMs (2 × 10^6^), LV-Sh H1299 cells (10^7^), LV-Sh H1299 cells (10^7^) and TAMs (2 × 10^6^). The cells were subcutaneously injected into the flanks of 6-week-old female nude mice. After 40 days, all mice were euthanized to excise the resultant tumors. We used the following formula to calculate the tumor volume: length × width^2^ / 2.

### Flow cytometry

We treated macrophages to prepare a single cell suspension and incubated with antibodies (PE Mouse anti-Human CD163, FITC Mouse anti-human CD11b, PC5.5 Mouse anti-human 7AAD, all from BioLegend, USA) at 4°C for 1 h. Next, we used flow buffer to wash cells twice, then centrifuged and resuspended them in 0.1 mL of the flow cytometry buffer for the analysis. We performed flow cytometry (Cytoflex, USA) and analyzed the results using Cytoflex software.

For the mouse model, we used collagenase digestion to obtain single-cell suspensions. The cells were then stained with fluorescence-labeled antibodies against F4/80, CD11b, and CD163 (BioLegend, USA).

### Statistical analysis

All data are expressed as mean ± standard deviation (SD). Statistical analysis was performed using GraphPad Prism 7, and one-way analysis of variance (ANOVA) was performed to determine significant differences between treatment groups. Differences between two groups were assessed using the Student's t-test, and P < 0.05 was considered to be statistically significant.

## Results

### Prognostic value and biological function of NEK2 in lung cancer patients based on bioinformatics

We downloaded RNA sequencing data from TCGA-LUAD samples (535 LUAD cancerous tissue samples and 59 adjacent noncancerous tissue samples). Under the threshold of FDA < 0.05, and |log2 FC| > 2, a total of 2,505 DEGs (1,977 upregulated and 528 downregulated in LUAD cancerous tissue samples) was identified. We first explored the correlation between the expression of the DEGs (Figure S1A). We noticed that high expression levels of NEK2 predicted the poor prognosis of LUAD patients (Figure 1A-D). To explore the function of NEK2 in LUAD, we carried out KEGG enrichment analysis and NEK2 single-gene GSEA analysis. The results showed that NEK2 was mainly enriched in the Wnt signaling pathway (Figure 1E) and participated in the process of macrophage polarization (Figure S1B). IHC was performed to detect NEK2 protein expression in the paired NSCLC tissues (Figure S1C). RT-qPCR was used to detect the expression of *NEK2* mRNA in a normal lung cell line and NSCLC cell lines (Figure S1D). The results showed that the expression of NEK2 in tumor cell lines or lung cancer tumor tissues was higher than that in the corresponding normal cells or neighboring normal tissues. These results indicated that NEK2 may be a potential biomarker for lung cancer.

### Loss of NEK2 inhibited cell proliferation and induced cell cycle arrest

To study the biological functions of NEK2, we selected 2 NSCLC cell lines, A549 and H1299, as models. We transfected non-specific control siRNAs (NC) and NEK2-specific siRNAs (si-1, si-2, and si-3) into A549 and H1299 cells. After 48 h treatment, to determine the knockdown efficiency of siRNAs, we detected the expression of *NEK2* mRNAs (Figure S2A). We chose 2 NEK2-specific siRNAs (si-1 and si-2) to test the protein levels of NEK2 (Figures S2B) and observed its effect on cell proliferation and cell cycle after the knockdown of NEK2. CCK-8 assay showed that, compared to the control group, the downregulation of NEK2 significantly inhibited cell proliferation. Furthermore, immunofluorescence and colony formation assays confirmed these results (Figure 2A-C and Figure S3). The results of flow cytometry showed that silencing of NEK2 blocked the cell cycle at the G0/G1 phase. The results of immunoblotting showed that NEK2 deficiency inhibited the expression of cell cycle-promoting proteins such as CDK2, CDK4, and CDK6 and promoted the expression of cell cycle-inhibiting proteins such as P21 and P27 (Figure 2D-E and Figure S4). These results indicated that NEK2 knockdown inhibited cell proliferation and cell cycle transition from G1 to S phase.

### NEK2 knockdown inhibited EMT of lung cancer cells through Wnt/β-catenin signaling pathway

When we performed wound healing assays (Figure 3A and B) and Transwell (Figure 3C-F) experiments in A549 and H1299 cells, we observed that NEK2 transfected with siRNA inhibited the migration and invasion of lung cancer cells. It is known that the classic Wnt/β-catenin signaling pathway is closely related to EMT. We analyzed EMT and Wnt/β-catenin signaling pathway-related molecules by immunoblotting (Figure 3G) and found that knocking down NEK2 effectively increased the expression levels of E-cadherin in A549 and H1299 cells. However, it reduced the levels of EMT-related proteins, such as MMP-9, Vimentin, and N-cadherin. At the same time, knockdown of NEK2 reduced the expression of β-catenin, c-Myc, and p-GSK3β (Ser9), but the expression of t-GSK3β remained unchanged. These results indicated that loss of NEK2 inhibited the migration and invasion of lung cancer cells through the Wnt/β-catenin signaling pathway.

### NEK2 acted as an oncogene in lung cancer cells

To conduct rescue experiments, we chose NEK2-specific siRNAs (si-1) as an example. A549 and H1299 cells were transfected with non-specific control siRNAs (NC), NEK2-specifific siRNAs (siRNA), and NEK2-specific siRNAs together with NEK2 overexpression plasmids (siRNA+OE). After 48 h treatment, the expression of *NEK2* mRNA was used to determine knockdown efficiency (Figure S5). We repeated some of the previous experiments, including CCK-8, immunofluorescence, colony formation related to cell proliferation, and wound healing assays, invasion, and migration related to EMT (Figure 4A-D and Figure 5A-F). At the same time, we also detected related molecules in EMT and the Wnt/β-catenin signaling pathway (Figure 5G). We found that NEK2 overexpression on the background of NEK2 knockdown alleviated changes in tumor cell biology caused by NEK2 knockdown. These results indicated that NEK2 promoted tumor progression.

### Knockdown of NEK2 inhibited M2 macrophages polarization in the lung cancer microenvironment

We used the supernatants of the NC and NEK2 knockdown groups to cultivate macrophages and observed changes in macrophage polarization. We tested whether the number of recruited macrophages and the cytokine secretion that caused M2-type polarization underwent changes after knocking down NEK2. The results of the Transwell assay showed that the number of recruited macrophages was reduced, and the mRNA levels showed that the expression level of *IL-10* was reduced (Figure 6A-C). Moreover, the concentration of IL-10 in conditioned media was tested by ELISA (Figure S6). The results were consistent with those of qRT-PCR. We then cultured M0 macrophages with supernatant of tumor cells, using RT-qPCR and flow cytometry to detect the changes in the surface markers and secretions of TAMs. We found that knocking down NEK2 reduced the expression of surface markers and secretion of M2-like macrophages (Figure 6D-F). Based on the RNA sequencing data provided in the TCGA database, the results suggested that NEK2 was positively correlated with the expression of IL10, and we verified the correlation at the protein level (Figure 6G-H). These results indicated that NEK2 knockdown inhibited the polarization of M2-like macrophages in the TME.

### Downregulation of NEK2 inhibited angiogenesis in lung cancer

To further explore the effects of NEK2 on angiogenesis, assays for angiogenesis and vascular endothelial cell migration experiments were conducted. The results confirmed that knocking down NEK2 inhibited blood vessel formation and vascular endothelial cell migration (Figure 7A-D). An analysis of the TCGA database suggested that NEK2 was positively correlated with vascular endothelial growth factor (VEGF) expression (Figure 7E). We verified the correlation at the mRNA and protein levels (Figure 7F-G). These results indicated that downregulation of NEK2 inhibited angiogenesis in the TME.

### NEK2 silencing inhibited lung cancer progression in a mouse model and changes the TME *in vivo*

To verify the effect of NEK2 on tumors *in vivo*, we used nude mice with lung cancer xenografts. H1299 LV-NC, H1299 LV-NC and TAMs, H1299 LV-Sh, H1299 LV-Sh and TAMs were injected subcutaneously into the right flanks of female nude mice. Tumors derived from H1299 LV-Sh cells were smaller and lighter in tumor volume and weight, respectively, than controls were, and TAMs could enhance the pro-tumor effects (Figure 8A-C and Figure S7). Additionally, flow cytometry showed that NEK2 knockdown resulted in a reduced ratio of 163+ M2 cells (Figure 8D and Figure S8), suggesting that NEK2 knockdown inhibited M2 polarization of macrophages. Immunohistochemical staining showed that NEK2 silencing attenuated the expression of NEK2, CD31, CD163, IL-10, Vimentin, and Ki67 in the xenografts (Figure 8E and Figure S9).

## Discussion

Some studies have shown that knocking down the *NEK2* gene played an important role in cancer treatment 31-33. However, the role of NEK2 in lung cancer is still unclear. By conducting a search in the GEPIA website, we found that the expression of NEK2 in lung cancer tissues was much higher than that in the adjacent tissues. A higher level of NEK2 expression indicated a poor prognosis. We asked whether NEK2 could promote the biological behavior of tumor cells, and to answer this question, we conducted a series of functional experiments. We found that silencing of NEK2 inhibited the proliferation of lung cancer cells, blocked the cycle in the G0/G1 phase, and inhibited EMT-related phenotypes such as invasion and migration.

The Wnt/β-catenin pathway is a canonical Wnt pathway, with β-catenin as the core protein. In normal mature cells, the Wnt/β-catenin signaling pathway is usually silent. However, in tumor cells, the Wnt/β-catenin pathway is aberrantly activated, participating in the occurrence and development of cancers by regulating cell cycle, cell proliferation, apoptosis, and cell adhesion 34-38. The Wnt signaling can upregulate the expression levels of Slug and Twist, which are transcriptional repressors of E-cadherin, thereby downregulating E-cadherin expression, resulting in the loss of intercellular adhesion and polarity, which is followed by EMT activation 39. In lung cancer, the Wnt/β-catenin signaling pathway also plays an important role. Animal experiments have shown that abnormal activation of the Wnt signaling pathway can lead to an increase in the incidence of primary lung cancer in experimental animals 40. The abnormal performance of the Wnt/β-catenin signaling pathway in lung cancer may be related to the abnormal expression or function of multiple components. Studies have shown that the expression of Wnt1 in surgically resected lung cancer tissues was significantly higher than that in the adjacent tissues 41. It has also been observed that the clinical prognosis in lung cancer patients with low expression of Wnt1, Wnt2, Wnt3, and β-catenin was better than that in the high expression group 41-43. In our results, we found that NEK2 could phosphorylate GSK, thereby promoting β-catenin to enter the nucleus and activating downstream factors such as c-Myc and CyclinD1, resulting in better proliferation, migration, and invasion abilities.

EMT is the driving force for malignant tumor cell migration and invasion, and it is a key molecular event in tumor metastasis 44, 45. The occurrence and metastasis in tumors and the formation of the TME are dynamic processes that involve interaction and mutual influence. EMT is initiated by hypoxia and inflammatory factors in the TME. In turn, EMT occurs in the TME and promotes tumor metastasis.

TAMs represent important components of the TME and are involved in tumor cell survival, proliferation, invasion, metastasis, survival, and prognosis. Macrophages stimulated by cellular interleukin-12, tumor necrosis factor-α, interferon-γ, bacterial lipopolysaccharide, Toll-like receptor agents, and pathogen-associated molecular patterns can be polarized to M1-type and play an important role in mediating T helper cell 1-type immune response and anti-pathogen infection 46, 47. IL-4, IL-5, IL-10, IL-13, colony-stimulating factor 1, transforming growth factor-β1, and prostaglandin E2 induce macrophages to M2-type polarization, which plays an important role in the process of tissue repair and remodeling 46, 48. In the past, it was believed that the main function of macrophages was to induce the body to produce immune responses through antigen presentation, thereby eliminating tumor cells or directly killing tumor cells. Therefore, macrophages play important roles in immune regulation against tumors. However, recent studies have shown that the infiltrating macrophages in the TME, that is, TAMs, cannot play an anti-tumor role; on the contrary, they promoted cancer progression and played a major role in the poor prognosis of cancer 27. In our study, we found that NEK2 knockdown inhibited the expression of IL-10, which induced macrophages to M2-type polarization.

Angiogenesis is the process of generating new blood vessels from existing endothelial cells to provide sufficient oxygen and nutrients to various organs. It is essential for the growth and metastasis of tumors and has been proven to be an important target for tumor treatment 49. Tumor angiogenesis is a complex process, which is strictly regulated by a variety of pro-angiogenic factors and anti-angiogenic factors. The key stimulating factor for angiogenesis in tumors is hypoxia, which promotes the excessive production of angiogenic factors such as VEGF. VEGF is the most important angiogenic factor. The VEGF family includes five glycoproteins VEGF-(A-E) and placental growth factors 1 and 2 50, 51. Most tumor cells express high levels of VEGF, which is often associated with poor tumor prognosis, risk of recurrence, disease progression, and low survival rate 52. Our research found that NEK2 knockdown inhibited the expression of VEGF and the process of tumor angiogenesis. Targeting NEK2 may reprogram the TME and improve the prognosis in lung cancer patients.

However, our study had some limitations. We have shown that NEK2 could lead to the polarization of macrophages and angiogenesis by affecting the secretion of IL-10 and VEGF, but we have not clarified how NEK2 changes the expression of IL-10 and VEGF. In addition, we did not rule out that NEK2 can affect the polarization of macrophages and tumor angiogenesis in other ways, which warrants further study.

In conclusion, our study is the first to demonstrate that NEK2 knockdown can deactivate the canonical Wnt/β-catenin signaling pathway in lung cancer cells, inhibites macrophage M2 polarization, angiogenesis, tumor growth, migration and metastasis. Therefore, targeting NEK2 may be a potential strategy for NSCLC therapy in the future.

## Supplementary Material

Supplementary figures and tables.

### Funding

This study was supported by the National Natural Science Foundation of China (81773236 and 81972852), Key Research & Development Project of Hubei Province (2020BCA069), Health Commission of Hubei Province Medical Leading Talent Project, Zhongnan Hospital of Wuhan University Science, Technology and Innovation Seed Fund (znpy2019048 and ZNJC201922), and Chinese Society of Clinical Oncology TopAlliance Tumor Immune Research Fund (Y-JS2019-036).

### Author contributions

Conghua Xie and Yan Gong contributed to the study design; Rui Bai and Cheng Yuan performed data collection and analysis; all authors contributed to manuscript preparation.

## Figures and Tables

**Figure 1:** ** Effect of NEK2 expression on survival and biological function in LUAD patients based on LUAD-TCGA data**. (A-D) Expression levels of NEK2 and the relationship between NEK2 and tumor stages, overall survival, and disease-free survival were investigated in the GEPIA database. (E) KEGG enrichment analysis suggests that NEK2 is enriched in the Wnt signaling pathway.

**Figure 2:** ** Downregulation of NEK2 suppressed NSCLC cell growth and survival *in vitro*.** (A) CCK-8 assays of A549 and H1299 cells transfected with NEK2 siRNAs or non-specific control siRNA. We measured the optical density (OD) values at 450 nm every 24 hours. (B) NEK2-specifific siRNAs (si-1 and si-2) inhibited colony formation of A549 and H1299 cells. (C) Immunofluorescence of Ki67 in A549 and H1299 cells transfected with NEK2 siRNAs or non-specific control siRNAs. Scale bar: 100 µm. (D) Flow cytometry shows the percentage of cells at different cell cycle phases. (E) After the cells were transfected with NEK2 siRNAs or non-specific control siRNAs, we conducted immunoblotting to analyze the cell cycle-related proteins in A549 and H1299 cells. Data are presented as mean ± SD of 3 independent experiments. *P < 0.05.

**Figure 3:** ** Knockdown of NEK2 inhibited the migration and invasion of lung cancer cells through Wnt/β-catenin signaling pathway.** (A-B) Representative photographs and quantification of wound healing assay of A549 and H1299 cells. Scale bar: 200 µm. (C-D) Representative photographs and quantification of transwell migration assays of A549 and H1299 cells. Scale bar: 100 µm. (E-F) Representative photographs and quantification of transwell invasion assay of A549 and H1299 cells. Scale bar: 100 µm. (G) The protein levels of EMT and Wnt/β-catenin pathway-related proteins were examined by immunoblotting. Data are presented mean ± SD of 3 independent experiments. *P < 0.05.

**Figure 4:** ** Rescue with NEK2 promoted cancer progression.** (A-B) The clone numbers of A549 and H1299 cells transfected with non-specific control siRNAs (NC), NEK2-specific siRNAs (siRNA) and NEK2-specific siRNAs with NEK2 overexpression plasmids (siRNA+OE) in colony formation assays. (C) CCK-8 assays in A549 and H1299 cells transfected with non-specific control siRNAs (NC), NEK2-specific siRNAs (siRNA) and NEK2-specific siRNAs with NEK2 overexpression plasmids (siRNA+OE). (D) Immunofluorescence of Ki67 in A549 and H1299 cells transfected with non-specific control siRNAs (NC), NEK2-specific siRNAs (siRNA) and NEK2-specific siRNAs with NEK2 overexpression plasmids (siRNA+OE). Data are presented as mean ± SD of 3 independent experiments. *P < 0.05.

**Figure 5:** ** Rescue with NEK2 promoted EMT of lung cancer cells.** (A-B) Quantification of wound healing assay of A549 and H1299 cells. Scale bar: 200 µm. (C-D) Representative photographs and quantification of transwell migration assays of A549 and H1299 cells. Scale bar: 100 µm. (E-F) Representative photographs and quantification of transwell invasion assays of A549 and H1299 cells. Scale bar: 100 µm. (G) The protein levels of EMT and Wnt/β-catenin pathway-related proteins were examined by immunoblotting. Data are presented as mean ± SD of 3 independent experiments. *P < 0.05.

**Figure 6:** ** Loss of NEK2 inhibited M2 macrophage polarization in lung cancer.** (A-B) Transwell migration uses THP-1 cells in the upper chamber and supernatants of transfected A549 and H1299 cells in the lower chamber. The average numbers of migrated cells are quantified. (C) We tested cytokines that can cause macrophage polarization secreted by A549 and H1299 cells transfected with NEK2 siRNAs or non-specific control siRNAs. (D) RT-qPCR detects changes in surface markers and secreted molecules in macrophages cultured with the supernatant of tumor cells. (E-F) Flow cytometry detects changes in surface markers in macrophages cultured with the supernatant of tumor cells. (G-H) The correlation between NEK2 and IL-10 based on TCGA (R2 = 0.254, P < 0.05) was verified at the protein levels. Data are presented as mean ± SD of 3 independent experiments. *P < 0.05.

**Figure 7:** ** Loss of NEK2 inhibited angiogenesis of lung cancer.** (A-B) Capillary tube formation of HUVECs incubated with conditioned medium from A549 and H1299 cells transfected with NEK2-specific siRNAs (si-1 and si-2) or non-specific control siRNAs (NC). (C-D) Transwell migration assays of HUVECs incubated with the conditioned medium from A549 and H1299 cells transfected with NEK2-specific siRNAs (si-1 and si-2) or non-specific control siRNAs (NC). (E-G) The correlation between NEK2 and VEGF based on TCGA (R2 = 0.373, P < 0.05) was verified by RT-qPCR and immunoblotting. Data are presented as mean ± SD of 3 independent experiments. *P < 0.05.

**Figure 8:** ** NEK2 knockdown inhibited lung cancer progression *in vivo*.** (A-B) Quantification of tumor volume and weight at 40 days after treatment. (C) After 40 days, the photos of tumors in H1299 LV-NC cells, H1299 LV-NC cells + TAMs, H1299 LV-Sh cells, H1299 LV-Sh cells + TAMs groups. (D) Flow cytometry detects the proportion of CD163+ M2 cells. (E) The expression of NEK2, CD163, IL-10, CD31, E-cadherin, Vimentin, and Ki67 in nude mouse tumor tissues is tested by immunohistochemistry. A heatmap was drawn using GraphPad. Data are presented as mean ± SD of 3 independent experiments. *P < 0.05.

## Abbreviations

TME: tumor microenvironment
TAMs: tumor-associated macrophages
NSCLC: non-small cell lung cancer
IHC: immunohistochemistry
